RETRACTED

# Effect of Proprioception and Balance Training Combined with Continuous Nursing on BBS Score and HSS Score of Patients Undergoing Total Knee Arthroplasty

**DOI:** 10.1155/2022/7074525

**Published:** 2022-07-01

**Authors:** Hong Lin, Aihua Xu, Heping Wu, Hanchun Xu, Yifang Lu, Hongping Yang

**Affiliations:** Department of Orthopedics, Hangzhou First People's Hospital, China

## Abstract

**Background:**

Total knee arthroplasty is one of the most effective methods for the treatment of end-stage knee osteoarthritis, but 10% of patients still show insufficient function, strength, and mobility. Continuous nursing service plays an important role in the rehabilitation of patients undergoing total knee arthroplasty. For discharged and convalescent patients, the traditional follow-up model cannot solve the nursing problems of discharged patients. How to meet the health needs of discharged patients under the limited nursing resources has become an existing problem.

**Objective:**

To explore the effect of proprioception and balance training combined with continuous nursing on Berg balance scale (BBS) score and Hospital for Special Surgery (HSS) score of patients undergoing total knee arthroplasty (TKA) is the objective of this study.

**Methods:**

Sixty patients undergoing TKA in our hospital from December 2019 to April 2021 were enrolled. The patients were randomly assigned into the control group and the study group. The control group received continuous nursing, and the study group received proprioception and balance training combined with continuous nursing.

**Results:**

The nursing satisfaction of the study group was higher than that of the control group (*P* < 0.05). The HSS scores at discharge, 1 month, 3 months, and 6 months after discharge in the study group were higher than those in the control group (*P* < 0.05). It was higher in the study group than in the control group at 1 month, 3 months, and 6 months after discharge (*P* < 0.05). The pain catastrophizing score of the study group at discharge was lower than that of the control group at 1 month, 3 months, and 6 months after discharge (*P* < 0.05). The BBS scores at discharge, 1 month, 3 months, and 6 months after discharge in the study group were higher than those in the control group (*P* < 0.05). The Lindmark balance scores at discharge, 1 month, 3 months, and 6 months after discharge in the study group were lower than those in the control group (*P* < 0.05).

**Conclusion:**

Proprioception and balance training combined with continuous nursing can effectively promote the recovery of knee joint function of patients after TKA, enhance patients' pain catastrophizing grade, enhance patients' quality of life, effectively promote patients' knee joint function and BBS score, and promote the improvement of disease.

RETRACTED

## 1. Introduction

Knee osteoarthritis (KOA) is a chronic degenerative disease characterized by degeneration of articular cartilage, subchondral sclerosis, reactive hyperplasia of articular margin, and subchondral bone [1]. It is the most common bone and joint disease in human limbs, and it is also the main cause of chronic pain and disability in adults. It affects about 250 million people worldwide, and the global prevalence rate is 3.8% [2]. The World Health Organization (WHO) lists it as an important factor affecting health status, which is one of the most common causes of disability in middle-aged and elderly patients [3]. At present, the pathogenesis of KOA is not clear, which may be related to age, obesity, inflammation, trauma, and genetic factors. It is most common in middle-aged obese women, whose main clinical manifestations are knee joint pain, swelling, deformity, and varying degrees of functional limitation [4]. As a progressive disease, it can lead to functional decline and life quality decline and has a huge impact on personal economy, health-care system, and social costs. TKA is one of the most effective methods for the treatment of end-stage KOA, which can effectively correct joint deformities, enhance joint function, and relieve joint pain [5]. About 90% of patients reported pain relief, improved functional ability, and life quality after TKA, but 10% of patients still indicated functional, strength, and mobility deficiencies [6]. At present, TKA is only an effective means to relieve the symptoms related to knee degenerative arthritis. Therefore, postoperative rehabilitation exercise has become an important measure to restore joint function [7].

In order to promote the sustainability of postoperative treatment and the effectiveness of rehabilitation exercise, we need to provide different forms of continuous nursing services for discharged patients to ensure the continuity of nursing services and the effectiveness of rehabilitation. In 1947, the concept of continuous care was first put forward in a research report in the USA [8]. The American Geriatric Association defines it as nursing intervention designed through a series of actions is a follow-up and extension of hospital nursing, which can help patients and their families complete the transition from hospital to family. High-quality, coordinated and continuous nursing measures are also available. Continuous nursing service plays a crucial role in the rehabilitation of patients after TKA. However, under current medical conditions, patients' needs for continuing care services are not being met effectively. The recovery of patients after TKA needs long-term and timely guidance from a professional medical team [9]. Whether the demand for continuous nursing service can be met is directly related to the recovery of joint function after operation. On the one hand, providing continuous nursing services can help patients deal with the disease effectively, enhance their compliance with rehabilitation exercise, reduce postoperative anxiety, relieve joint pain, and promote the rehabilitation process of patients after TKA. On the other hand, understanding the needs of patients after TKA is very important for clinical nurses to make relevant continuous nursing programs [10]. However, the contradiction between the growing demand for health care and the uneven distribution of health resources is difficult to change in the short term. Health-care workers often focus on inpatients. For the discharged and convalescent patients, the traditional follow-up model cannot solve the nursing problems of discharged patients. How to meet the health needs of discharged patients with limited nursing resources has become an existing problem [11].

RETRACTED

In the field of sports training, neuromuscular training represented by balance training is often adopted to optimize sports performance, prevent injury, or provide rehabilitation [12]. Some studies have indicated that these training interventions have a positive impact on reducing the risk of sports injury and can promote the functional performance after sports injury [13]. It is pointed out that the changes of proprioceptive sensation and neuromuscular control are the main reasons of these effects [14]. Keitkamp et al. have indicated that balance training can significantly increase the standing time of one leg on the unstable interface, but strength training cannot enhance it [15]. Meanwhile, balance training can increase the maximum contractile strength of knee flexion and extension under isokinetic condition. On the other hand, Taube et al. indicated that after 6 weeks of balance training, the maximum contractile strength of lower limbs did not change significantly, nor did its strongest development rate, nor did it change significantly during the maximum contraction of soleus, gastrocnemius, tibialis anterior, quadriceps, and biceps femoris. Some studies have also suggested that balance training cannot significantly improve sports performance compared with super-isometric training [16]. It is found that the knee muscle strength, vertical jump height, and posture control are enhanced, but there exhibits no significant difference [17]. In this regard, Astrid et al. pointed out that the effects of balance training on vertical jump and sensitive performance are still controversial, but balance training may have a positive impact on these sports performance [18]. Many scholars have studied the effects of balance training, the combination of balance training and strength training, and the combination of balance training and explosive power training on sports performance [19]. However, these training based on experiments are interfered by all kinds of trainings. Some scholars define neuromuscular training as a multiple intervention system composed of balance training, strength training, stretching-contraction exercises, agility training, and special exercises [20]. Therefore, it is not clear whether a single training intervention is the fundamental factor affecting the training results or the whole intervention system. Moreover, many theories believe that balance training can promote the proprioceptive sensation of the body, and it is generally evaluated by changing the body posture under one's own weight, such as one-foot balance [21]. Balance training has been indicated to strengthen human stability, but the effect on specific joint proprioceptive sensation is not clear. The Hospital for Special Surgery (HSS) score which was proposed by the American Hospital in 1976 consists of the following six parts: pain (30 points), function (22 points), range of motion (18 points), muscle strength (10 points), knee flexion deformity (10points), and stability (10 points). When the patients walk with the help of the crutches or there is varus deformity or valgus deformity in their knee joints, these points will be reduced accordingly. HSS scoring system 6 emphasizes pain, function, and range of motion, which is well known for its high degree of interobserver correlation. The Berg balance scale (BBS) score was used to evaluate the patient's balance function, including 14 related activities, such as sitting station transfer, unsupported standing, and unsupported sitting. The higher the score, the better the balance function. Based on this, this study focuses on the effect of proprioception and balance training combined with continuous nursing on BBS score and HSS score of patients undergoing TKA.

RETRACTED

## 2. Patients and Methods

### 2.1. General Information

Sixty patients undergoing TKA in our hospital from December 2019 to April 2021 were enrolled. The patients were randomly divided into the control group and the study group. The control group received continuous nursing, while the study group received proprioception and balance training combined with continuous nursing. In the control group, the age was 43-74 years old with an average age (65.66 ± 3.53), including 18 males and 12 females, while in the study group, the age was 44-76 years old with an average of age (65.68 ± 3.56), including 16 males and 14 females. There exhibited no statistical significance in the general data. This study was permitted by the Medical Ethics Association of our hospital, and all patients signed informed consent.

Inclusion criteria are as follows: (1) unilateral or bilateral TKA and in accordance with TKA indications; (2) the age was18-85 years old; and (3) patients and their families agreed to participate in this study and sign an informed consent form.

Exclusion criteria are as follows: (1) patients who accompanied by severe organ dysfunction, malignant tumors, and rare diseases and (2) patients with mental disorders, consciousness disorders, and cognitive disorders.

### 2.2. Treatment Methods

The control group received continuous nursing, and the WeChat platform continuous nursing group was established. According to TKA disease management, a continuous nursing team was set up, which was composed of deputy chief nurse, attending physician, rehabilitation therapist, and 3 competent nurses. The head nurse was adopted as the team leader to train the members on nursing-related contents after TKA. The day before the patient's discharge, the nursing staff instructed the patients to follow and use the WeChat platform to ensure that the patients and their families were proficient in the operation. (1) TKA disease knowledge is posted once a week, with content edited by team members according to patient needs. Other links are copied and reviewed by the deputy chief nurse and sent by the postgraduate nursing students in the form of text and pictures and videos. The contents of releases include TKA-related knowledge, medication instruction, rehabilitation functional exercise instruction, dietary instruction, disease monitoring, psychological instruction, and follow-up visits. (2) Patients can watch video instructions through the “functional exercise” module to carry out effective and correct functional exercise. (3) Patients can conduct self-evaluation in the “investigation tools” module. (4) The nursing graduate students count the results of knee joint function, quality of life, and pain catastrophizing level self-tested on WeChat platform and inform the deputy chief nurse patients' scores every month. (5) By adding WeChat friends, group members can provide personalized help according to the needs of different patients. Patients with poor self-evaluation can be urged to exercise through voice chat and video chat to promote the recovery.

The study group received proprioception and balance training combined with continuous nursing, and the continuous nursing was the same as that of the control group. The specific measures of proprioceptive and balance training are as follows: (1) standing exercise: arm chair back and foot exercise “one foot exercise” (bipedal exercise requires the center of gravity to change between healthy feet), 20 times in each group, 5 times a day for two weeks; (2) balance instrument two-foot center of gravity control training, to find the center of gravity displayed on the screen, 5 groups a day, practice for 1 week; and (3) balance instrument single-foot center of gravity control training, 5 groups a day, practice for 1 week.

RETRACTED

### 2.3. Observation Index

#### 2.3.1. Satisfaction

By consulting the literature and expert discussion, the patient follow-up satisfaction was designed; a total of 10 items were designed to record the patient's satisfaction with the follow-up management mode, health education, medical and nursing service, and appointment registration process. It is divided into four dimensions: very satisfied, relatively satisfied, general satisfied, and dissatisfied. Satisfaction rate = very satisfaction rate + relatively satisfaction rate + general satisfaction rate.

#### 2.3.2. Knee Joint Function Score

Hospital for Special Surgery (HSS) score is a scale compiled by Insall et al. to evaluate knee joint function in patients with TKA. The scale consists of 7 questions, of which 6 items are scored items (pain, joint function, range of motion, muscle strength, flexion deformity, and joint stability), and 1 item is deducted, including the need for walker, incomplete extension, and valgus deformity, and the total score is 100. The score ≤59 indicates poor knee joint function, 60~69 is general, 70~84 is good, and ≥85 is excellent. The higher the score, the better the knee function. In this study, the Cronbach's *α* coefficient of the scale was 0.910.

#### 2.3.3. Concise Health Survey Scale

The Mos 36-item Short Form Health Survey (SF-36) is a Chinese version of the scale translated by Li Lu et al. to evaluate the quality of life of patients with TKA. The scale includes physical health and mental health. The physical health includes three dimensions: physiological function, physical pain, and general health. The mental health includes four dimensions: energy, social function, emotional function, and mental health. The scale consists of 36 items. The final score of each dimension = (actual score-the lowest possible score in this area)/the difference between the highest score and the lowest score in this area ×100; the score range of each dimension is from 0 to 100; the higher the score, the better the quality of life. In this study, the Cronbach's *α* coefficient of the scale was 0.908.

RETRACTED

#### 2.3.4. Pain Catastrophizing Scale

Pain catastrophizing scale (PCS) is a Chinese version of the pain catastrophizing scale (PCS) written by Yap et al. It is adopted to evaluate the pain catastrophizing level of patients with TKA. The scale includes three dimensions of helplessness, exaggeration, and repeated consideration with a total of 13 items. From “never” to “always like this,” the total score is 0.52. The score ≥38 indicates that the pain degree reaches the level of pain catastrophizing. In this study, the Cronbach's *α* coefficient of the scale is 0.968.

#### 2.3.5. Berg Balance Scale

Berg balance scale (BBS), which can be employed to evaluate the balance function of the subjects under dynamic and static conditions, can also be adopted to predict the possibility of falls under normal conditions. The following points indicate that there is a risk of falling: 0-20 points: poor balance ability, which means patients can only sit in a wheelchair; 20-40 points: balance ability, which means patients can assist walking; and 41-56 points: good balance ability, which means patients can walk independently.

#### 2.3.6. Lindmark Balance Score

The Lindmark balance score includes standing independently, sitting alone, standing on one leg, standing on one leg, etc. The highest score for each item is 15. The higher the score, the stronger the patient's balance response ability.

### 2.4. Statistical Analysis

SPSS 22.0 statistical analysis software was employed to analyze the following: (1) Descriptive analysis: measurement data and semimeasurement data are expressed by (symptom score) as $\bar{x}\pm \text{s}$ count data rate or composition (ratio); (2) hypothesis testing: parametric and nonparametric tests were employed, respectively; and (3) specific methods: *t*-test is employed for measurement data in accordance with normal distribution (correction *t*-test is used when variance is uneven); Mann–Whitney *U* test is adopted for nonnormal distribution (MmurW test); measurement data are tested by MmurW test with nonparametric correlation or independent samples; nongrade counting data are tested by *χ*2 test; grade count data are tested by Ridit test; significance test level *a* = 0.05; and *P* < 0.05 indicates that the difference exhibits statistically significant.

## 3. Results

### 3.1. Comparison of Nursing Satisfaction

First of all, we compared the nursing satisfaction: The study group was very satisfied in 20 cases, satisfactory in 7 cases, and general in 3 cases; the satisfaction rate was 100.00%; the control group was very satisfied in 13 cases, satisfactory in 9 cases, general in 4 cases, and dissatisfied in 4 cases; and the satisfaction rate was 86.67%. The nursing satisfaction of the study group was higher than that of the control group (*P* < 0.05). All the data results are indicated in Figure 1.

RETRACTED

### 3.2. HSS Score Comparison

Secondly, we compared the HSS scores. Before nursing, there exhibited no significant difference (*P* > 0.05). After nursing, the HSS score increased. The HSS score of the study group at discharge was higher than that of the control group at 1 month, 3 months, and 6 months after discharge (*P* < 0.05). All the data results are indicated in Figure 2.

### 3.3. Comparison of Life Quality Scores

Thirdly, we compared the scores of life quality. Before nursing, there exhibited no significant difference (*P* > 0.05). After nursing, the score of life quality increased. With regard to the score of life quality at discharge, 1 month, 3 months, and 6 months after discharge in the study group were higher compared to the control group (*P* < 0.05). All the data results are indicated in Figure 3.

### 3.4. Comparison of the Scores of Pain Catastrophizing

Then, we compared the pain catastrophizing scores. Before nursing, there exhibited no significant difference (*P* > 0.05). After nursing, the pain catastrophizing score decreased. Next, the pain catastrophizing score of the study group at discharge, 1 month, 3 months, and 6 months after discharge was lower compared to the control group (*P* < 0.05). All the data results are indicated in Table 1.

### 3.5. BBS Score Comparison

Next, we compared the BBS score. Before nursing, there exhibited no significant difference (*P* > 0.05). After nursing, the BBS score increased. In terms of the BBS score of the study group at discharge, 1 month, 3 months, and 6 months after discharge were higher compared to the control group (*P* < 0.05). All the data results are indicated in Table 2.

### 3.6. Lindmark Balance Score Comparison

Finally, we compared the Lindmark balance score, and before nursing, there exhibited no significant difference (*P* > 0.05). After nursing, the Lindmark balance score increased. Regarding the Lindmark balance score of the study group at discharge, 1 month, 3 months, and 6 months after discharge were higher compared to the control group (*P* < 0.05). All the data results are indicated in Table 3.

## 4. Discussion

KOA has become a worldwide disease affecting the health of the middle-aged and elderly, which is one of the main causes of disability in the elderly [10]. At present, TKA is considered to be an effective surgical method for the treatment of severe KOA, which can relieve knee joint pain, correct joint deformity, and enhance dysfunction. A great deal of evidence shows that rehabilitation after TKA is useful, but maintaining effective therapeutic effect is still a challenge [11]. Therefore, we need to develop more flexible and personalized treatment plans to promote the sustainability of postoperative treatment. Continuous care should be given when returning to the family [12]. In the following decades, with the rapid development of the global economy and the reform of the medical service system, the goal of effectively shortening the duration of hospitalization was put forward, and more people were discharged without full recovery. This leads to a higher demand for nursing after discharge [13]. Patients hope that medical staff can continue to provide continuous and coordinated nursing services after discharge and urge them to complete their recovery at a later stage. The concept of continuous care came into being in this environment to ensure that different patients enjoy continuous and coordinated care during referrals [14]. Therefore, the western developed countries, led by the USA, began to attach importance to the development of continuous nursing services for patients after discharge, formulated a series of systematic continuous nursing programs and put them into practice, and achieved good clinical results. It laid the foundation for further nursing research. Subsequently, scholars from various countries have also carried out extended nursing research one after another, and their definitions are not the same [15]. So far, the concept of continuous care has not been uniformly defined. At present, it is defined by the American Geriatric Association in 2003: Nursing intervention designed through a series of actions is the follow-up and extension of hospital nursing, which can help patients and their families complete the transformation from hospital to family. High-quality, coordinated, and continuous nursing measures are also available [16]. In the 1980s, Naylor and others organized an intervention study on continuous nursing. The results indicated that continuous nursing model based on family follow-up could effectively enhance the prognosis of patients. It was a low-cost and effective nursing model, and it was the earliest research on continuous nursing [17]. With the implementation of health and medical management standards, in order to reduce the average days of hospitalization, promote patient turnover, and increase the use of medical resources, more patients are discharged early without full recovery [18]. The data has indicated that in recent years, anesthetic techniques, a variety of analgesic treatments, perioperative medical optimization, and surgical techniques have greatly shortened the length of stay after TKA, but reducing the average length of stay is still continuing to improve management [19]. Some literatures have indicated that the recovery effect of TKA is related to regular and standardized functional exercise after operation [20]. Patients may need more personalized and adaptive information and continuous nursing services of doctors, nurses, and rehabilitators after discharge [21].

RETRACTED

This study found that the nursing satisfaction of the study group was higher than that of the control group (*P* < 0.05). The HSS scores at discharge, 1 month, 3 months, and 6 months after discharge in the study group were higher than those in the control group (*P* < 0.05). It was higher in the study group than in the control group at 1 month, 3 months, and 6 months after discharge (*P* < 0.05). The pain catastrophizing score of the study group at discharge was lower than that of the control group at 1 month, 3 months, and 6 months after discharge (*P* < 0.05). The BBS scores at discharge, 1 month, 3 months, and 6 months after discharge in the study group were higher than those in the control group (*P* < 0.05). The Lindmark balance scores at discharge, 1 month, 3 months, and 6 months after discharge in the study group were lower than those in the control group (*P* < 0.05), which suggested that proprioception and balance training combined with continuous nursing can effectively promote the recovery of knee joint function of patients after TKA, improve the level of pain catastrophizing, enhance the quality of life of patients, effectively promote knee joint function and BBS score, and promote the recovery of knee joint function of patients. We believe that the reason is that balance is the process of maintaining the position of the body's center of gravity perpendicular to the support, relying on fast and continuous feedback from visual, vestibular, and somatosensory structures, and then performing smooth and coordinated neuromuscular movements [22]. The balance ability of human body is mainly divided into static balance and dynamic balance. Static balance refers to the ability of the human body to maintain the center of gravity and control the relative stillness of body posture. When the body is still, the body cannot be completely still. The weight of the body moves around its own balance point and is not controlled by self-consciousness, which is called physiological posture jitter [23]. Dynamic balance refers to the ability of the human body to adjust and control the center of gravity and posture during exercise. Human dynamic balance involves the sensitivity of receptors, the afferent pathways of information, the integration of centers, and the comprehensive properties of neuromuscular efferent pathways. Balance training has been adopted to promote balance and exercise-related skills, as well as the prevention and rehabilitation of lower limb sports injuries. The main areas are involved in the rehabilitation of patients with diseases and sports injuries, the improvement of balance ability of the elderly, and the development of athletes' physical ability and related sports skills [24]. Studies have indicated that patients with cervical spondylosis, hemiplegia, brain trauma, stroke, osteoporosis, spinal cord compression, Parkinson's disease, multiple sclerosis, and their dynamic balance ability will decline in varying degrees. In the rehabilitation training to cure these diseases, balance training is often adopted as the main means of rehabilitation. Gunes and other studies have indicated that biofeedback training with computer balancer can strengthen the posture control and weight support of hemiplegic patients when walking [25]. However, Ruth's results were different from most studies, and his experiments did not find that biofeedback training significantly improved the balance ability of stroke patients [26]. However, Ruth also pointed out that due to the small sample size of his observation, further research should be carried out. The application of balance training in the prevention and rehabilitation of sports injuries is mainly focused on the prevention and rehabilitation of ankle and knee joint injuries. Trojian et al. carried out single leg balance test (SLB) on athletes and found that there was a significant negative correlation between ankle injury and single leg balance test results [27]. Emery pointed out that in the study of college students and senior high school students, balance training was helpful to prevent the occurrence of sports injuries. After summarizing the previous studies, Jessica et al. said that balance training can prevent the injury of anterior cruciate ligament of knee joint [28]. However, there is not a systematic balance training method for clinical design to prevent sports injury. Proprioceptive perception is the sensation produced by proprioceptors by sensing the dynamic and static states of the body and joints, which can be summarized as joint position perception and motion perception in clinic. There are three aspects: reflex response and muscle tone regulation. The effect of meniscus injury on the proprioceptive sensation of the knee joint is mainly reflected in the loss of proprioceptor after the injury that weakens the ability of afferent and efferent motor signals and then affects the proprioceptive sensation of the knee joint [29]. Proprioceptive neuromuscular facilitation therapy (PNF) enhances the neuromuscular response and promotes muscle contraction by using motor and positional stimuli. Its main purpose is to enhance the motility, stability, control ability of joints, and the skills of how to complete compound movements [29, 30]. For example, the brain adjusts the stride length through the signals sent out by proprioceptive sensation, so as to maintain the accuracy of motion and position perception. Jiang Yongjun carried out the balance promotion training for patients with ACL injury reconstruction and pointed out that balance promotion training could significantly improve the recovery of knee joint proprioceptive ability of patients after ACL injury reconstruction [30–32]. As a way to prevent acute ankle injury and chronic ankle instability, balance training is widely used in ankle rehabilitation. Verhagen and others have conducted balance board training for professional volleyball players and pointed out that it can significantly reduce the incidence of ankle injury and reinjury [33]. Guine and other studies also supported this point of view. Their randomized controlled trials on balance training of ankle injuries point out that balance training can significantly reduce the incidence of ankle injuries [34].

RETRACTED

In summary, proprioception and balance training combined with continuous nursing can effectively promote the recovery of knee joint function of patients after TKA, enhance patients' pain catastrophizing level, strengthen patients' quality of life, and effectively facilitate patients' knee joint function and BBS score, promoting the improvement of the disease.

## Figures and Tables

**Figure 1:** Comparison of nursing satisfaction between two groups.

**Figure 2:** Comparison of HSS scores between two groups of patients. Note: compared with the control group, ∗*P* < 0.05.

**Figure 3:** Comparison of patients' quality of life scores between two groups. Note: compared with the control group, ∗*P* < 0.05.

**Table 1:** Comparison of pain catastrophizing scores between the two groups ($\bar{x}\pm \text{s}$, points).

Group	*N*	Before nursing	When discharged from the hospital	One month after discharge	3 months after discharge	6 months after discharge
C group	30	43.91 ± 1.66	35.76 ± 3.78	29.49 ± 5.63	20.84 ± 3.31	14.81 ± 3.31
S group	30	43.77 ± 1.65	32.59 ± 3.31	24.91 ± 2.56	15.53 ± 4.31	6.78 ± 4.12
*t*		0.327	3.455	4.056	5.351	8.322
*P*		>0.05	<0.01	<0.01	<0.01	<0.01

**Table 2:** Comparison of BBS score between the two groups ($\bar{x}\pm \text{s}$, points).

Group	*N*	Before nursing	When discharged from the hospital	One month after discharge	3 months after discharge	6 months after discharge
C group	30	6.48 ± 2.43	7.06 ± 1.21	10.69 ± 3.34	16.44 ± 3.31	23.12 ± 3.44
S group	30	6.41 ± 2.56	8.92 ± 1.34	16.84 ± 3.11	22.77 ± 3.31	34.67 ± 2.44
*t*		0.108	5.642	7.380	7.406	14.999
*P*		>0.05	<0.01	<0.01	<0.01	<0.01

RETRACTED

**Table 3:** Comparison of Lindmark balance score between the two groups ($\bar{x}\pm \text{s}$, points).

Group	*N*	Before nursing	When discharged from the hospital	One month after discharge	3 months after discharge	6 months after discharge
C group	30	5.78 ± 1.44	6.57 ± 1.45	8.44 ± 1.22	9.49 ± 1.24	10.74 ± 1.22
S group	30	5.67 ± 1.24	8.18 ± 2.11	10.92 ± 1.22	12.59 ± 1.23	14.15 ± 0.21
*t*		0.317	3.444	7.872	9.721	15.087
*P*		>0.05	<0.01	<0.01	<0.01	<0.01

## Data Availability

The simulation experiment data used to support the findings of this study are available from the corresponding author upon request.
